# Application of Deep Learning Technology in Predicting the Risk of Inpatient Death in Intensive Care Unit

**DOI:** 10.1155/2021/6169481

**Published:** 2021-12-01

**Authors:** Ming Li, HuiLin Chen, ShuYing Yan, Xiao Xu, HuaJuan Xu

**Affiliations:** Shanghai Jiangong Hospital Intensive Care Unit (ICU), Shanghai 200083, China

## Abstract

The Intensive Care Unit (ICU) is an important unit for the rescue of critically ill patients in hospitals, and patient mortality is an important indicator to measure the level of ICU treatment. Currently, a variety of clinical scoring systems are used to evaluate the patient's condition and predict survival, but these systems require a lot of resources. However, due to the rapid development of artificial intelligence and deep learning, machine learning based methods have been used to study the survival prediction of ICU patients. Additionally, these methods have made significant progress, but there is still a distance from clinical application, and equally metric interpretability of the deep learning method is not very mature. Therefore, in this paper, we have proposed a predicting model for the life and death of ICU patients, which is primarily based on the Fuzzy ARTMAP model. With a thorough analysis of the existing ICU patient condition assessment and life and death prediction methods, we have observed that patient's ICU monitoring information performs integrated analysis and extracts features according to the clinical characteristics of physiological indicators. Finally, fuzzy ARTMAP neural network is used to predict the life and death of patients. Likewise, prediction results are combined with the clinical scoring system and logistic regression, artificial neural network, support vector machine, and AdaBoost. Experimental results of these algorithms were compared, which verifies that the proposed method has outperformed the existing model. The main purpose of the proposed mode is to design a life and death prediction method for ICU patients, which has high predictive performance and is an acceptable method for clinical medical staff, where ICU monitoring data is used. Experimental results show that the method proposed has achieved better prediction performance and accuracy ratio, which provide theoretical reference for clinical application.

## 1. Introduction

Critical Care Medicine is a discipline that studies the laws and characteristics of the development process of the human body to death caused by various injuries or illnesses and treats critically ill patients according to these laws and characteristics. Its purpose is to achieve centralized treatment of critically ill patients, thereby reducing the input of medical resources, improving the level of hospital treatment, and reducing the mortality of critically ill patients. With the establishment of the intensive care unit and its important role in medical work, intensive care medicine has now become an indispensable part of our country's medical system. In order to promote the research and development of critical care medicine in our country, in July 2008, the National Standardization Administration approved the establishment of critical care medicine as a secondary discipline of clinical medicine [1].

The ICU is a specialized department in the hospital that focuses on monitoring and treating critically ill patients. It can provide timely standardized and high-quality medical monitoring and treatment techniques to patients whose organ and system dysfunction caused by various factors are life-threatening or potentially highly dangerous. The ICU applies the most cutting-edge diagnostic, monitoring, and treatment instruments and technologies to conduct uninterrupted, real-time quantitative and qualitative observations of patients' disease conditions, and through effective treatment measures, to provide patients with more effective and high-level life support, improves the quality of life of patients [2]. There are many clinical methods and standards for evaluating the treatment level and service quality of ICU. One of the important indicators is the effective evaluation of critically ill patients and the effective prediction of their prognostic status.

Patients entering the ICU usually have multiple organs and system dysfunctions. In order to fully understand and analyze the patient's condition and potential risks, doctors need to collect different physiological indicators of the patient, which are constantly changing compared with the basic information of the patient. The physiological indicators can better reflect the criticality of the patient's condition. Because the physiological indicators collected by each patient are sequential and diverse, each patient generates a large amount of high-dimensional and complex physiological data during ICU treatment. How to analyze the massive physiological data of the patient and extract the hidden value from it is studied. Meaningful information has become a hot and difficult problem in the current medical field and data mining field [3–5].

At present, different scoring systems are commonly used in medicine to evaluate the severity of critical illnesses and predict the mortality of ICU patients. These scoring systems can provide clinical decision-making support for medical staff to a certain extent. Due to the incompleteness of experience treatment knowledge and the massiveness of ICU monitoring data, data errors are prone to occur in the scoring process, leading to distortion of the evaluation results and huge labor costs. Therefore, in the context of the rapid development of information technology and artificial intelligence, the use of data mining and machine learning methods for ICU data analysis and patient condition prediction has become a research hotspot in recent years.

The life and death prediction research of ICU patients is significant. First, accurate life and death predictions for ICU patients can improve the survival probability of critically ill patients; secondly, early life and death predictions for ICU patients, as a useful indicator to measure the medical level, can help doctors evaluate the patient's condition and objectively formulate and revise medical care plans. To determine the best time to leave the hospital and reduce overtreatment of patients, thereby reducing the cost of treatment for patients, again, accurate prediction of the life and death of ICU patients is conducive to evaluating the effects of medical measures and doctors' work and improving the quality of medical care; finally, it is also reasonable to configure ICU medical resources that play an important role in creating a good doctor-patient relationship.

Due to the diversity and complexity of the physiological data of ICU patients, the use of the traditional critical illness scoring system to deal with the life and death prediction of ICU patients can no longer meet the clinical needs of the ICU. In recent years, the combination of ICU patient life and death prediction problems with data mining knowledge has become a new way to solve the problem. Through the improvement and optimization of traditional prediction methods, massive medical data is studied with the help of machine learning algorithms, combining the advantages of different algorithms. The improvement of the algorithm and the construction of the model are used to decompose the complex problems and finally realize the patient's condition assessment and life and death prediction.

In this paper, we have proposed a predicting model for the life and death of ICU patients, which is primarily based on the Fuzzy ARTMAP model. With a thorough analysis of the existing ICU patient condition assessment and life and death prediction methods, we have observed that patient's ICU monitoring information performs integrated analysis and extracts features according to the clinical characteristics of physiological indicators. Major research features of the proposed model are given as follows:

- Development of a Fuzzy ARTMAP model based patient life and death prediction system for patients admitted to the ICU unit in hospital.
- A mechanism that has the capacity to thoroughly evaluate existing ICU patient's data in the hospital.
- Development or implementation of the clinical scoring system, which further enhances the accuracy and prediction ratio of the proposed model.

The rest of the paper is managed according to the following format.

In section-2, existing state-of-the-art methods are extensively evaluated, in addition to how these models are not capable of addressing the problem under consideration in this paper.

## 2. Related Work

At present, clinical evaluation of patients' condition and life and death prediction are mainly carried out through a scoring system. The scoring system is weighted or assigned according to the important symptoms, signs, and physiological parameters of the disease to quantify the severity of critical illness [6]. Currently, widely used scoring systems include Acute Physiology and Chronic Health Status Score System (APACHE), Concise Acute Physiological Function Score System (SAPS), Sequential Organ Failure Score System (SOFA), and Death Probability Model (MPM) [7–11]. Among them, APACHE and SAPS scoring systems are commonly used in ICU. In actual clinical application, because the APACHE II scoring system has good predictive ability on the condition and prognosis of critically ill patients, it has become the most widely used disease evaluation system in the field of ICU at home and abroad. Xu et al. [12] found that the APACHE II score predicted mortality rate was significantly higher than the actual mortality rate; Park et al. [13] found that the predicted mortality rate was higher than the actual mortality rate in neurosurgery ICU. Jin et al. [14] found that the APACHE II score is very valuable for assessing the life and death of critically ill patients in internal medicine and surgery, but it is not suitable for predicting the life and death of patients with cardiovascular disease. Liu et al. [15] and others found that the APACHE II scoring system also has limitations in obstetric applications. After the advent of the APACHE scoring system, Le Gall et al. proposed a simple scoring system, the SAPS scoring system. The SAPS scoring system is a perfection to the APACHE scoring system. Compared with the APACHE scoring system, the physiological indicators it uses are in clinical practice. It is easier to collect, and there is no need to consider the patient's diagnosis when predicting the condition. The clinical use is more convenient. The evaluation found that the SAPS scoring system has a higher prediction accuracy than the APS score [16–20], which can be used as a simpler one, and the time-saving method is used for comparative research and management evaluation between different ICUs. The common feature of the above-mentioned scoring system is that the corresponding scores are given according to the scores of the scoring table according to the physiological indicators and physical signs of the patients, and then the critical condition of the patients is judged according to the scores. At the same time, the death risk prediction formula is used from the perspective of probability. Calculate the risk of the patient. The scoring system has undergone many iterations and improvements over the years, but the changes and improvements of the scoring system are mainly manifested in the impact of parameter items in the scoring table, parameter score weights, patient admission time on the accuracy of disease prediction, and death risk prediction adjustment and correction of the coefficients in the formula.

The characteristic of data mining is to be able to discover its implicit internal connection and value information in a large amount of chaotic data. The progress and development of artificial intelligence and the complexity and massiveness of ICU monitoring data make people think of applying data mining knowledge to the life and death prediction study of ICU patients. The application of machine learning methods in medical data mining can effectively improve the efficiency and quality of medical data mining. Therefore, in recent years, the use of machine learning methods to study the life and death prediction of ICU patients has become a development trend. In 2012, the MIT Computational Physiology Laboratory held an international competition based on machine learning for ICU patient life and death prediction algorithms. They provided the ICU physiological parameter data of 4000 patients including 4 different ICU types and gave the prediction results of the SAPS scoring system as a comparison.

Hamilton et al. [21] used the stepwise regression method to select 40 variables from the PhysioNet data set as the independent variables of the logistic regression model, and the patient outcome (life or death) was used as the dependent variable for prediction. Bera et al. [22] selected 30 parameters and took the maximum, average, and minimum values of each time series plus age, a total of 88 parameters, as the input variables of the logistic regression model. Macas et al. [23] proposed using a linear Bayesian classifier to study the life and death prediction problem of ICU patients. Through preprocessing and correlation analysis, some unestimable parameters were used to train the linear Bayesian classifier with the feature vector after dimensionality reduction. Johnson et al. [24] proposed a Bayesian ensemble scheme composed of 500 weak learners to predict the life and death of ICU patients. Each weak learner is a two-depth decision tree, which can randomly assign an intercept and slope to a randomly selected single feature, and the parameters of the learner set are determined by Markov chain Monte Carlo sampling. Xia et al. [25] proposed the use of artificial neural network methods to study the life and death prediction of ICU patients. The trend parameters of the time series constructed by linear regression together constitute a 141-dimensional feature vector. Pollard et al. [26] used a combination of physical analysis methods used to discover solar nanoflares and artificial neural networks to predict the life and death of ICU patients. Finally, the conjugate gradient BP network is used to classify the features. Citi et al. [27] used the cascaded support vector machine-generalized linear model paradigm to study the life and death prediction of ICU patients and normalized the variables. Bosnjak et al. [28] proposed the use of statistics and support vector machines to study ICU patient condition prediction. However, the results show that the method has overfitting problems, and the prediction results are not ideal. Taylor et al. [29] extracted more than 500 clinical data variables from patients' electronic health records to construct a random forest model and used the model to predict the mortality of patients. Churpek et al. [30] used a large, multicenter database to study the accuracy of patient clinical deterioration prediction.

## 3. Realization of Life and Death Prediction System for the ICU Patients

In this section, a detailed description of the ICU patient life and death prediction method, which is based on Fuzzy ARTMAP neural network, is presented and discussed in detail. The experiment content mainly includes three parts: data preprocessing, feature extraction, and prediction realization. The prediction framework is shown in Figure 1.

### 3.1. Fuzzy ARTMAP Neural Network

Neural network is based on the knowledge of network topology, simulating the processing mechanism of the human brain's nervous system to complex information, and expressing complex functional relationships through a large number of simple relationship connections. Among the many neural network models, the fuzzy ARTMAP neural network has been favored by the majority of researchers because of its good predictive performance. It combines the methods of adaptive resonance theory (ART) and fuzzy mathematics theory. It not only has fast and stable online recognition learning ability and high-quality resolution, but also has good operability. In recent years, it has received extensive attention from the research community.

#### 3.1.1. Adaptive Resonance Theory

Adaptive Resonance Theory (ART) was proposed by Grossberg. Subsequently, Grossberg and Carpenter et al. conducted in-depth research on ART and proposed an important ART neural network model in 1988 [31]. After years of research and continuous development, the ART model has three forms: ARTl, ART2, and ART3. ART is a self-organizing neural network. It is an unsupervised, vector clustering and competitive learning classification algorithm based on behavior and cognitive models. It can self-organize any number and complexity of two-dimensional inputs, as well as stable and large-scale parallel processing. ART is a self-organizing classification algorithm that imitates the logical cognitive process of the human brain. It shows unique advantages in the face of modern increasingly complex data classification. The main advantages of the ART model are as follows: (1) it is a real-time online learning and can adapt to the dynamic environment; (2) it has a stable and rapid recognition of the learned patterns and can quickly adapt to new content; (3) it has the ability of self-normalization, and according to the situation, some features are sometimes used as key features, and sometimes treated as noise; (4) it is unsupervised learning, and the storage capacity is not affected by other attributes. The ART model is based on the basic idea of a competition-cooperative network interaction model. The model is shown in Figure 2.

We have observed that the competition-cooperative network 1 is simultaneously affected by the signals from the environment input and the top-down learning results; among them, the bottom-up learning is not only the output of the competition-cooperative network 1, but also the output of the competition-cooperative network 2. The output of competition-cooperative network 2 is top-down learning. The final result is produced through the continuous learning and matching of this network. The environmental input signal stimulates the top-down learning result, so that the competition-cooperative network 1 outputs a bottom-up learning result. The competition-cooperative network 2 receives the input, generates a top-down learning result output, and returns to the competition-cooperative network 1. This process is a top-down learning process and a bottom-up learning process, and there is a steady stream of environmental input signals in this process. Through the learning and matching of competition-cooperative network, the final result is obtained. However, this kind of competitive learning network has the disadvantage of unstable classification, that is, the appearance of a new one.

The emergence of ART model successfully resolved the competition. It addresses the problem of unstable classification in the cooperative network model. The ART model adds a stabilizing mechanism to the simple competitive learning model. The short-term memory STM and long-term memory LTM are added to the competitive learning mechanism to ensure that the original memory content is not lost. Under the premise of destruction, new memory content can be added to the model to achieve the purpose of real-time online learning, so as to overcome stability.

#### 3.1.2. Fuzzy Theory

Many things and phenomena in the real world do not have clear concepts, but people can understand these things and phenomena heartily and rarely cause misunderstanding and ambiguity. These phenomena that cannot be accurately described because there is no strict boundary division are called fuzzy phenomena, and various concepts that reflect fuzzy phenomena are called fuzzy concepts. Fuzzy theory is a science developed to solve the ubiquitous fuzzy phenomena in the real world. Fuzzy theory is developed on the mathematical basis of fuzzy set theory founded by Professor Zadeh of the University of California in 1965. Fuzzy sets are the basis of fuzzy theory. The basic idea of fuzzy theory is to accept and agree with the existence of fuzzy phenomena, with the goal of solving vague and uncertain objects, and try to convert them into content that can be processed by computers.

Professor Zadeh first proposed a new tool to express the ambiguity of things in 1965, namely, the membership function. By using the membership function to express the fuzzy concept, it can give a quantitative expression to the fuzzy concept. The proposal of membership function breaks through the classic set theory, thus laying a good mathematical foundation for fuzzy theory. The emergence of the membership function breaks the limitation that the membership degree of the element to the set in the classic set can only be 0 or 1. It can be extended to any value in the interval [0, 1], which makes the problem of description ambiguity more reasonable.

#### 3.1.3. Fuzzy ARTMAP

Fuzzy ARTMAP neural network is an incremental supervised learning mode that can make multidimensional response and classification recognition to any dimensional analog input vector. It realizes the combination of fuzzy theory and adaptive resonance theory mapping [32] by using the close similarity between fuzzy subset calculation and ART in learning, resonance, and classification selection. Not only that, fuzzy ARTMAP also corrects the prediction error by increasing the minimum threshold of ART's alert parameter during the matching and tracking process, thereby realizing a new maximum and minimum learning rule to maximize the minimum prediction error and maximize compression coding. It can meet the accuracy standard requirements by automatically learning the minimum number of classification categories or hidden units.

Fuzzy ARTMAP is a network structure that combines ARTMAP neural network and fuzzy theory. It can make stable online learning and classification prediction for any input mode. The structure of fuzzy ARTMAP is shown in Figure 3:

For the ART system, the *F*_0_ node in each ART system represents the current input vector; the *F*_1_ node accepts the bottom-up vector from *F*_0_ and the activation code or classification output from *F*_2_ from top to bottom. The number of nodes in *F*_0_, *F*_1_ and *F*_2_ is arbitrary. Among them, the input vector of *F*_0_ is expressed as

(1) $$\begin{array}{c} I=\left(I_{1},\ldots ,I_{M}\right). \end{array}$$

The activation vector of *F*_1_ is expressed as

(2) $$\begin{array}{c} X=\left(x_{1},\ldots ,x_{M}\right). \end{array}$$

The activation vector of *F*_2_ is expressed as

(3) $$\begin{array}{c} Y=\left(y_{1},\ldots ,y_{M}\right). \end{array}$$

The adaptive weight or LTM tracking vector of each *F*_2_ category node is expressed as

(4) $$\begin{array}{c} \omega_{j}=\left(\omega_{j1},\ldots ,\omega_{jM}\right). \end{array}$$

where *j* represents the category node of *F*_2_, the initial value represents that each category is unconstrained, and the representation is

(5) $$\begin{array}{c} \omega_{j1}\left(0\right)=\cdots =\omega_{jM}\left(0\right)\\ =1. \end{array}$$

For each input vector *I* and *F*_2_, the decision function is defined as

(6) $$\begin{array}{c} T_{j}\left(I\right)=\frac{\left|I\wedge \omega_{j}\right|}{\alpha +\left|\omega_{j}\right|}, \end{array}$$

where *ω*_*j*_ is the weight vector of the j-th node, *α* is the decision parameter, and ∧ is the concept of fuzzy as follows:

(7) $$\begin{array}{c} \left(p^{q}\right)=\text{min}\left(p,q\right). \end{array}$$

When the search is completed, the weight vector will be updated according to the following formula:

(8) $$\begin{array}{c} \omega_{J}^{\text{new}}=\beta \left(I\wedge \omega_{J}^{\text{old}}\right)+\left(1-\beta \right)\omega_{J}^{\text{old}}. \end{array}$$

### 3.2. Data Preprocessing

The physiological indicators in the experimental data have varying degrees of missing, and the missing of these data will not only make the data incomplete and affect the effective use of the experimental data, but also cause deviations in the subsequent predictive experimental results. Therefore, it is particularly important to adopt an effective and high-quality method to deal with the problem of missing data.

Three data preprocessing methods for missing data will be used below, namely, normal value filling method, mean value filling method, and binary filling method, to fill and organize the experimental data set. The process framework of the three data preprocessing methods is shown in Figure 2. It can be seen that the processing steps of the three data preprocessing methods are to first organize and summarize the physiological index data recorded by each patient to construct a data matrix of physiological indexes, then construct a matrix of filling data according to the filling method, and then use the filling matrix fill in the missing data of patients; finally, the complete physiological index matrix of each patient is merged into the physiological index matrix of all patients. Among them, the biggest difference lies in the data selection and matrix generation methods of the data filling matrix. Each data filling method will be introduced in Figure 4.

#### 3.2.1. Normal Value Filling

The main idea of this method is to use the normal range of physiological indicators to fill in the missing data of physiological indicators. The filling steps are as follows: (1) convert the physiological index record file of each patient into the cell matrix of the corresponding physiological index; (2) extract a random value from the normal range of each physiological index to construct a filling matrix; (3) judge the cell array of each physiological index in the cell matrix. If it is empty, find the corresponding filling value in the matrix to fill it to form a new cell matrix; (4) the cell matrix composed of complete physiological indicators of each patient is combined to form a cell matrix of physiological indicators of all patients. The above steps constitute the physiological index matrix of all patients in this method.

#### 3.2.2. Mean Filling

The main idea of this method is to fill in the average value of the physiological index of all patients of the same sex in the age group of the patient according to the age of the patient and then fill in the missing physiological index record of the patient. The filling steps are as follows:

1. Convert the physiological index record file of each patient into a cell matrix of the corresponding physiological index.
2. Group the ages of all patients, and calculate the average value of each physiological index according to gender for each group of patients. The male patient is constructed into a filled matrix, and the female patient is constructed into a filled matrix.
3. The cell array of each physiological index in the cell matrix is judged. If it is empty, find the physiological index filling value of the corresponding age in the matrix of the same gender as the patient. Fill in to form a new cell matrix.
4. Combine the cell matrix composed of the complete physiological indicators of each patient to form a cell matrix of the physiological indicators of all patients. The above steps constitute the physiological index matrix of all patients in this method.

#### 3.2.3. Binary Filling

The main idea of this method is to change the physiological index with a degree of missing more than half to 0 or 1. If a physiological index has a record of monitoring data, then the recorded value of the physiological index is filled with 1, indicating that the physiological index and these indicators are documented. If there is no record of monitoring data for a certain physiological index, the record of this physiological index is filled with 0, which means that the physiological index has no record. For the physiological indicators whose degree of absence does not exceed half, the values in the normal range are used for filling. The filling steps are as follows:

1. Convert the physiological index record file of each patient into a cell matrix of the corresponding physiological index.
2. Judge the physiological index in the matrix, and determine the physiological index that is missing more than half according to whether there is a record set of this item to 1 or 0, and the rest remain unchanged.
3. Extract a random value from the normal value range of each physiological index to construct a filled matrix.
4. For each physiological index in the cell matrix, cell array is judged. If it is empty, find the corresponding filling value in the matrix and fill it to form a new cell matrix.
5. Combine the cell matrix composed of the complete physiological index of each patient to form the physiological index of all patients cell matrix. The above steps constitute the physiological index matrix of all patients in this method.

### 3.3. Feature Extraction

The feature extraction of ICU patient monitoring data is a key link in predicting the life and death of ICU patients. The feature extraction determines the accuracy and efficiency of the prediction to a large extent. Through effective feature extraction methods, the accuracy of the prediction results can be improved. After data preprocessing, complete physiological indicators of all patients are obtained, but what is obtained is a cell matrix of high-dimensional physiological indicator data. The structure of this matrix is more complicated, and each cell array contains one or more physiological indicators. The value and structure are irregular, so the regular feature matrix used in the subsequent prediction research should be extracted from this matrix. Based on the clinical significance of the physiological data of ICU patients, this study will select some indicators from the data set as the characteristics of this experiment. The extracted feature matrix includes three parts. The first part is the basic information characteristics of ICU patients, including the patient's age, gender (0 means female, 1 means male), and ICU type (1: Cardiac Intensive Care Unit, 2: Cardiac Surgery Rehabilitation Ward, 3: Internal Medicine Intensive Care Unit, 4: Surgical Intensive Care Unit) three basic information; the second part is the 36 physiological index characteristics monitored after the patient is admitted to the ICU, and the minimum and average values are extracted for each physiological index value and the maximum values are three items of data. The third part is the life and death status of the patient when leaving the ICU (0: survival, 1: death). After the above feature extraction steps, the irregular data matrix is preliminarily processed into a regular backup feature matrix. Enter the fuzzy ARTMAP model to predict life and death.

## 4. Experiments and Discussion

### 4.1. Datasets

The data set used in this study contains data from four different types of ICU wards, namely, coronary care unit, cardiac surgery rehabilitation unit, medical intensive care unit, and surgical intensive care unit. The data set contains a total of 4000 clinical data of ICU patients. Among them, there are 577 cases (14.43%) in the coronary care unit, and 874 cases (21.85%) in the cardiac surgery rehabilitation ward. There are 1481 patients in the intensive care unit (37.03%), and 1068 patients (26.70%) in the surgical intensive care unit. There are 3446 surviving cases (accounting for the total) of the 4000 patient cases, 86.15% of the number of cases, and 554 deaths (13.85% of the total number of cases). All the cases were adults over 16 years old, and the time spent in ICU was more than 48 hours. During the first 48 hours of admission, each patient recorded a maximum of 42 items of information, including 6 items of basic patient information and 36 dynamic monitoring data of physiological indicators [33].

### 4.2. Evaluation Metrics

TP represents the predicted death of the patient and the actual death, FP represents the predicted death, but the actual outcome is survival, FN represents the predicted survival, but the actual death, and the TN predicted survival and actual survival. Sensitivity *S*_*e*_ refers to the percentage of actual deaths that are correctly identified as deaths based on the predicted results of the research; specificity refers to the percentage of actual survival that is correctly identified as survivals based on the predicted results of the research; precision *P* refers to the percentage of deaths that are actually predicted as deaths percentage; accuracy refers to the ratio of the number of patients who correctly predict the life and death of patients to all patients. In this study, the smaller value of sensitivity and accuracy, namely, min(*S*_*e*_, *P*), will be used to evaluate the prediction effect of the prediction model.

### 4.3. Evaluation on Different Filling Methods

In order to verify the impact of the three data preprocessing methods proposed in this article on the prediction results, the following will initially use the fuzzy ARTMAP neural network to predict the effects of the three data preprocessing methods: normal value filling method, mean value filling method, and binary filling method. Test and experiment to verify each method by 5 times of 10-fold cross-validation experiments. The following will describe the experimental results of each scheme separately, which is shown in Tables 1, 2, 3 and 4.

It can be seen from Tables 1–4 that the experimental results obtained by using the binary filling method have a poor overall prediction effect; although the experimental results obtained by the normal value filling method fluctuate greatly, the prediction effect is generally better than the other two methods. According to the analysis of the above experimental results, the characteristic matrix formed by the data processed by the normal value filling method can better reflect the clinical characteristics of the physiological indicators of ICU patients, and the prediction effect is better. Therefore, this study will use the normal value filling method to solve the lack of ICU data. At the same time, the characteristic matrix formed by the data filled by this method is used as the matrix for subsequent research.

### 4.4. Comparison with Existing Methods

On the basis of verifying the effects of the three data preprocessing methods, in order to further verify the prediction effect based on the Fuzzy ARTMAP model, this study compares the experimental results with the prediction results of other methods using the same data set in the literature (SAPS [34], ANN [25], SVM [28], Logistic Regression [35], and AdaBoost [36]). The study will compare the average prediction accuracy with other methods. The prediction results are shown in Table 5.

It can be seen that the prediction results of different methods using the same data set in the existing literature are different, and the differences are large. Among them, the clinical SAPS scoring system has the worst prediction effect, and the prediction result based on the cascade AdaBoost model is the best. Although the life and death prediction results of ICU patients based on fuzzy ARTMAP neural network proposed in this study are not optimal, they still show good prediction results. Through the above comparison, the feasibility of the method proposed in this study is verified.

## 5. Conclusions

In this paper, we analyzed advantages and disadvantages of existing models and combined the characteristics of ICU clinical monitoring data to propose a method for predicting the life and death of ICU patients, which is based on the fuzzy ARTMAP model. Although this method is compared with existing research methods, its predictive effect is not optimal, but the main advantage is that fuzzy ARTMAP can not only obtain stable prediction results, but also obtain easy-to-understand interpretation rules, which is helpful for clinical medical staff to understand and accept the prediction results. The main contributions of this paper are as follows: (1) we summarize and analyze the existing ICU patient life and death prediction research methods and their advantages and disadvantages, so as to provide guidance and reference for the design of the research methods in this paper. (2) Three data preprocessing methods are designed. By sorting out the patient's experimental data and analyzing its characteristics, three methods for processing missing data, namely, normal value filling, mean value filling, and binary filling, are proposed, and the data processed by the three methods are extracted, respectively. According to the physiological significance of the ICU clinical monitoring data, the basic information of the patient, the minimum, average and maximum values of physiological indicators, and the life and death status are used to form the characteristic matrix of ICU patients. (3) N uses fuzzy ARTMAP neural network to verify the effect of three data preprocessing methods. By comparing the prediction effects of the three methods, the effectiveness of the data preprocessing method using normal value filling is determined. After comparing the prediction results of the model with the prediction results of other machine learning methods, the effectiveness of the prediction method based on the fuzzy ARTMAP model is confirmed.

## Figures and Tables

**Figure 1:** Framework of Prediction based on Fuzzy ARTMAP.

**Figure 2:** Competition-cooperation network interactive model.

**Figure 3:** Structural diagram of fuzzy ARTMAP.

**Figure 4:** Flow chart of data filling methods.

**Table 1:** Prediction results of filling method with normal value.

Item	*S*_*e*_	*P*	min(*S*_*e*_, *P*)
1	73.86	65.11	65.11
2	51.59	63.78	51.59
3	67.38	66.01	66.01
4	63.77	54.08	54.08
5	61.49	65.13	61.49
Ave	63.62	62.82	59.66

**Table 2:** Prediction results of filling method with mean value.

Item	*S*_*e*_	*P*	min(*S*_*e*_, *P*)
1	56.08	67.09	56.08
2	47.54	71.34	47.54
3	71.33	59.01	59.01
4	65.98	58.31	58.31
5	51.24	57.25	51.24
Ave	58.43	62.60	54.44

**Table 3:** Prediction results of filling method with binary value.

Item	*S*_*e*_	*P*	min(*S*_*e*_, *P*)
1	68.55	45.31	45.31
2	58.69	53.19	53.19
3	54.98	48.87	48.87
4	50.15	60.13	50.15
5	40.17	62.94	40.17
Ave	54.51	54.10	47.54

**Table 4:** Evaluation on different filling methods.

Method	*S*_*e*_	*P*	min(*S*_*e*_, *P*)
Normal	63.62	62.82	59.66
Mean	58.43	62.60	54.44
Binary	54.51	54.10	47.54

**Table 5:** Prediction results with different methods.

Method	min(*S*_*e*_, *P*)
SAPS	30.54
ANN	48.87
SVM	52.57
Logistic regression	55.08
Fuzzy ARTMAP	59.66
AdaBoost	78.56

## Data Availability

The datasets used and analyzed during the current study are available from the corresponding author upon reasonable request.

## References

[1] Liu D. (2011). Development of critical care medicine in China. *Chinese Journal of Practical Internal Medicine*.

[2] Wang H., Cao W. (2012). Features and requirements of intensive care unit (ICU). *Chinese Community Doctors*.

[3] Wu X., Liu C., Wang L., Bilal M. (2021). Internet of things-enabled real-time health monitoring system using deep learning. *Neural Computing & Applications*.

[4] Pei J. (2020). Big data mining in the control of epidemic. *Basic and Clinical Pharmacology and Toxicology*.

[5] Zhong K., Wang P., Pei J. (2021). Multi objective optimization regarding vehicles and power grids. *Wireless Communications and Mobile Computing*.

[6] Li S., Zhang Q., Xie C. (2012). Progress in the severity scoring system of patients in adult intensive care unit. *Chinese Journal of Primary Medicine and Pharmacy*.

[7] Gong N., Li Q. (2015). Research progress of common critical illness scores in clinical application. *Journal of Youjiang Medical University for Nationalities*.

[8] Knaus W., Zimmerman J. E., Wagner D. P., Draper E. A., Lawrence D. E. (1981). Apache-acute physiology and chronic health evaluation: a physiologically based classification system. *Critical Care Medicine*.

[9] Knaus W., Draper E., Wagner D. (1986). Apache II: a severity of disease classification system. *Critical Care Medicine*.

[10] Knaus W. A., Wagner D. P., Draper E. A. (1991). The Apache III prognostic system. *Chest*.

[11] Zimmerman J. E., Kramer A. A., Mcnair D. S. (2006). Acute Physiology and Chronic Health Evaluation (Apache) IV: hospital mortality assessment for today’s critically ill patients∗. *Critical Care Medicine*.

[12] Xu W., Fang L., Liu L. (2010). Analysis of the value of Apache II score and SAPS II score in predicting mortality in critically III patients. *Chinese Journal of Hemorheology*.

[13] Park S., Chun H., Kim D. (2009). Acute physiology and chronic health evaluation II and simplified acute physiology score II in predicting hospital mortality of neurosurgical intensive care unit patients. *Journal of Korean Medical Science*.

[14] Jin S. (2005). Clinical application of Apache score in critically ill patients. *Hebei Medical Journal*.

[15] Liu H., Wang Q., Xu Z. (2005). Application of acute physiology and chronic health evaluation II for critically ill obstetric patients admitted to GICU. *Chinese Journal of Clinical Obstetrics and Gynecology*.

[16] Pei J., Li J., Zhou B., Bin Z., Gao M., Dat Q. A recommendation algorithm about choosing travel means for urban residents in intelligent traffic system.

[17] Gall J., Loirat P., Alperovitch A. (1984). A simplified acute physiology score for ICU patients. *Critical Care Medicine*.

[18] Barlage S., Gnewuch C. (2009). Changes in HDL-associated apolipoproteins relate to mortality in human sepsis and correlate to monocyte and platelet activation. *Intensive Care Medicine*.

[19] Lu S., Li Y., Wu L. (2015). Application and progress of Apache scoring system. *Military Medical Journal of Southeast China*.

[20] Pei J. Solving the problem of charging and discharging of electric vehicles based on particle swarm algorithm.

[21] Hamilton S., Hamilton J. Predicting in-hospital-death and mortality percentage using logistic regression.

[22] Zhang M. (2021). Applications of deep learning in news text classification. *Scientific Programming for Smart Internet of Things*.

[23] Macas M., Kuzilek J., Odstrcilik T. Linear bayes classification for mortality prediction.

[24] Johnson A., Dunkley N., Mayaud L., Tsanas A., Kramer A. A., Clifford G. D. Patient specific predictions in the intensive care unit using a bayesian ensemble.

[25] Xia H., Daley B., Petrie A., Zhao X. A neural network model for mortality prediction in ICU.

[26] Pollard T., Harra L., Williams D., Harris S., Martinez D., Fong K. PhysioNet Challenge: an artificial neural network to predict mortality in ICU patients and application of solar physics analysis methods.

[27] Citi L., Barbieri R. PhysioNet 2012 Challenge: predicting mortality of ICU patients using a cascaded SVM-GLM paradigm.

[28] Bosnjak A., Montilla G. Predicting mortality of ICU patients using statistics of physiological variables and support vector machines.

[29] Taylor R. A., Pare J. R., Venkatesh A. K. (2016). Prediction of in-hospital mortality in emergency department patients with sepsis: a local big data-driven, machine learning approach. *Academic Emergency Medicine*.

[30] Churpek M. M., Yuen T. C., Winslow C. (2016). Multicenter comparison of machine learning methods and conventional regression for predicting clinical deterioration on the wards. *Critical Care Medicine*.

[31] Carpenter G., Grossberg S. (1998). The ART of adaptive pattern recognition by a self-organizing neural network. *Computer*.

[32] Carpenter G., Grossberg S., Reynolds J. (1991). ARTMAP: supervised real-time learning and classification of nonstationary data by a self-organizing neural network. *Neural Networks*.

[33] Moody G. B., Mark R. G. (2001). PhysioNet: a Web-based resource for the study of physiologic signals. *IEEE Engineering in Medicine and Biology Magazine*.

[34] Le Gall J. R., Lemeshow S., Saulnier E. (1993). A new Simplified Acute Physiology Score (SAPS II) based on a European/North American multicenter study. *Journal of the American Medical Association: The Journal of the American Medical Association*.

[35] Marco L., Bojamejad M., King S. T. Robust prediction of patient mortality from 48 hour intensive care unit data.

[36] Yi C., Sun Y., Tian Y. CinC Challenge: predicting in-hospital mortality in the intensive care unit by analyzing histograms of medical variables under Cascaded Adaboost model.

